The article "Tree bark scrape fungus: A potential source of laccase for application in bioremediation of non-textile dyes" was retracted in 2025. Reasons: a conflict of interest; concerns about the results or conclusions; concerns about the peer review; concerns about the authorship.

# Tree bark scrape fungus: A potential source of laccase for application in bioremediation of non-textile dyes

**DOI:** 10.1371/journal.pone.0229968

**Published:** 2020-06-04

**Authors:** R. Z. Sayyed, H. M. Bhamare, Sapna, Najat Marraiki, Abdallah M. Elgorban, Asad Syed, Hesham Ali El-Enshasy, Daniel J. Dailin

**Affiliations:** 1 Department of Microbiology, PSGVP Mandal’s Arts, Science and Commerce College, Shahada, India; 2 Department of Biotechnology, SSVP Sansth’s Late Karmveer Dr. P. R. Ghogrey Science College, Dhule, India; 3 ICAR-National Bureau of Plant Genetic Resources, New Delhi, India; 4 Department of Botany and Microbiology, College of Science, King Saud University, Riyadh, Saudi Arabia; 5 Centre of Excellence in Biotechnology Research, King Saud University, Riyadh, Saudi Arabia; 6 Institute of Bioproduct Development, Universiti Teknologi Malaysia (UTM), Skudai, Johor Bahru, Malaysia; 7 School of Chemical and Energy Engineering, Faculty of Engineering, Universiti Teknologi Malaysia (UTM), Skudai, Johor Bahru, Malaysia; 8 City of Scientific Research and Technology Applications, New Burg Al Arab, Alexandria, Egypt; North Eastern Regional Institute of Science and Technology, INDIA

## Abstract

Although laccase has been recognized as a wonder molecule and green enzyme, the use of low yielding fungal strains, poor production, purification, and low enzyme kinetics have hampered its large-scale application. Thus,this study aims to select high yielding fungal strains and optimize the production, purification, and kinetics of laccase of *Aspergillus* sp. HB_RZ4. The results obtained indicated that *Aspergillus* sp. HB_RZ4 produced a significantly large amount of laccase under meso-acidophilic shaking conditions in a medium containing glucose and yeast extract. A 25 μM CuSO_4_ was observed to enhance the enzyme yield. The enzyme was best purified on a Sephadex G-100 column. The purified enzyme resembled laccase of *A*. *flavus*. The kinetics of the purified enzyme revealed high substrate specificity and good velocity of reaction,using ABTS as a substrate. The enzyme was observed to be stable over various pH values and temperatures. The peptide structure of the purified enzyme was found to resemble laccase of *A*. *kawachii* IFO 4308. The fungus was observed to decolorize various dyes independent of the requirement of a laccase mediator system.*Aspergillus* sp. HB_RZ4 was observed to be a potent natural producer of laccase, and it decolorized the dyes even in the absence of a laccase mediator system. Thus, it can be used for bioremediation of effluent that contains non-textile dyes.

## Introduction

Laccase (benzenediol: oxygen oxidoreductase, EC 1.10.3.2), belonging to a group of enzymes called multicopper blue oxidasehas been noted to exhibit a wide substrate specificity [1]. It has been applied in various sectors, such as biomedical [2], dye degradation [3], paper industries for delignification [4–5], bioremediation [6], in biosensors [7], as melanin degraders in the cosmetic industry [8], as an enzymatic biofuel [9] and used in juice clarification [10]. Furthermore, laccase is a key biological mediator and the best alternative for chemical mediators; thus, it is regarded as a green enzyme in dye degradation, which is a new era for dye degradation [11]. Synthetic dyes are broadly used in a wide range of industries, including textiles, paper, printing, cosmetics, and pharmaceuticals. During dyeing, 10–15% of the dyes are lost in the effluent. Owing to their structural complexity, most of these dyes resist biodecolorization [12]. Although physic-chemical approaches are available for the removal of these dyes, they have found to be costly and non-eco-friendly [12].

High catalytic efficiency is another key feature of the enzyme that has been utilized in the bioremediation of dye effluent, sulfonamide, and other pollutants. This bioremediation ismediated by thelaccase mediator system (LMS) [13]. Laccase has emerged as a significant enzyme in the mycoremediation of grey-water treatment as it substantially reduces the chemical oxygen demand (COD) and biological oxygen demand (BOD), and solids present in grey-water [14]. The new trend of forward osmosis, aided by laccase, is used in the removal of micro-pollutants from wastewater and increase the potability of water [15]. Laccase is also used in the biodegradation of organics, as it is a critical factor in reducing water pollution with its excellent catalytic performance and reusability [16,17].

Laccase has a self as well as a cross-coupling mechanism for catalyzing single-electron oxidation, playing an important role in removing non-degradable organic pollutants [18]. It is now used as an effective and best alternative for chemical bleaching agents,which are used for paper bleaching in the paper industry [19]. Nonetheless, high production cost and low efficiency of laccase has restricted its wider application and has increased the need to develop an economically feasible process [20]. The production yield of an enzyme depends on the type of producing strain, as most natural strains are known to be poor laccase producers. However, screening and selecting potent laccase producing fungi and optimizingthe production conditions continue to remain crucial and vital approachesto achieving high and cost-effective yields of laccase. Furthermore, improvement in laccase production by optimizing medium composition and cultivation parameters has been reported [21].

## Materials and methods

### Chemicals

All the chemicals used in this study were purchased from Hi-media laboratories, India;and Remazol Brilliant Blue R and 2,2’-azino-bis(3-ethylbenzothiazoline-6-sulphonic acid) (ABTS) were procured from Sigma Aldrich, USA.

### Source of culture

*Aspergillus* sp. HB_RZ4 used in this study was obtained from the Department of Biotechnology, SSVPS’s Science College, Dhule, Maharashtra, India. It was previously isolated from tree bark scraping [22].

### Screening for laccase production

In this study, three different media, namely tannic acid agar [23], guaiacol agar (GuA), and gallic acid agar (GAA), containing 0.5% tannic acid, 3% malt extract, and 0.5% mycological peptone, respectively, were used to screen the production of ligninolytic enzymes. In GuA and GAA, tannic acid was replaced with guaiacol (0.01%) and gallic acid (0.5%), respectively. One plug (1 cm indiameter) of *Aspergillus* sp. HB_RZ4 culture was grown on each plate at 32 °C for 6 d andsubsequently observed for the formation of brown halos around the fungal growth.

Alternatively, one plug (1 cm in diameter) of *Aspergillus* sp. HB_RZ4 was grown at 32 °C for 5 d on selective basal media plates containing (gL^-1^) peptone, 3.0; glucose, 10.0; KH_2_PO_4_, 0.6; ZnSO_4_, 0.001; K_2_HPO_4_, 0.4; FeSO_4_, 0.0005; MnSO_4_, 0.05; MgSO_4_, 0.5; and agar 2%, supplemented with 0.1% (w/v) ABTS [24].

### Production of laccase

For laccase production,two plugs of fungus were grown at 32 °C for 12 d in aminimal medium (MM) containing (gL^-1^) glucose, 3.0; KH_2_PO_4_, 1.0; (NH_4_)_2_SO_4_, 0.26; MgSO_4_.7H_2_O, 0.5; CuSO_4_.7H_2_O, 00.5; 2,2-dimethyl succinic acid, 2.2; CaCl_2_.2H_2_O, 0.74; ZnSO_4_.7H_2_O, 0.6; FeSO_4_.7H_2_O, 0.5; MnSO_4_.4H_2_O, 0.5; CoCl_2_.6H_2_O, 0.1; and a 0.50 μl vitamin solution with4.5 pH [25]. Afterwards, the medium was centrifuged at 10,000 rpm for 15 min at 4 °C to obtain a cell-free extract, which was subsequently used for laccase assay,using ABTS as the standard (100–1000 μgmL^-1^) [26].

### Laccase assay

The reaction mixture, comprising of 2.0 ml 100 mM sodium acetate buffer (pH 4.0), 80 μl ABTS, and 20 μl enzyme, was incubated for 10 min [27] and the oxidation of ABTS was later recorded at 420 nm (εmax = 36000 M^-1^cm^-1^) and expressed in units per ml (UmL^-1^). One unit of the enzyme was defined as the enzyme required for the formation of one μM of the product per min [28, 29].

### Estimation of fungal growth

Afterincubation, the MM was filtered through a Whatman filter paper No l, and the resultant biomass was dried at 70°C and weighed till a constant weight was achieved, which was expressed in mgmL^-1^.

### Optimization experiments

Cultural conditions and media variables for optimum growth and production of laccase were optimized using theOne Variable at a Time (OVAT) approach.

#### Influence of incubation period on the growth and production of laccase

To ascertain the exact time for the optimum growth and production of laccase, two plugs of fungalgrowth of 1cm diameter each were grown in a basal medium for 12 d at 32 °C and120 rpm [24]. The samples were withdrawn after every 24 h and were subsequently examined for estimatingthe laccase activity and fungal growth.

#### Optimization of variables for growth and production of laccase

The physical parameters, for example,pH (2–10), temperature (20–55°C), incubation time (1–12 d) [24], and nutrients, such as carbon sources (1.5%),which included glucose, sucrose, starch, maltose, lactose, fructose, and glycerol, organic nitrogen sources (1.5%), such as L-asparagine, glutamic acid, glycine, L-proline, yeast extract, peptone, urea, inorganic nitrogen sources (1.5%),which includedammonium nitrate, sodium nitrate, potassium nitrate, ammonium chloride, ammonium dihydrogen phosphate, and ammonium sulfate, inducers (10–50 μM), namely CuSO_4_, tween 80, veratryl alcohol, guaiacol, 2,5 xylidine, vanillic acid, gallic acid, ammonium tartrate, and vanillin were optimized forthemaximumproduction of laccase [30].

### Purification of enzyme

The cell-free extract of the production medium was precipitated with ammonium sulfate, in a concentration range of 10–85% (w/v), under continuous stirring at 4 °C. Afterward, the precipitate was separated through centrifugation,with a centrifugal force of 5,000×g for 10 min at 4°C and re-dissolved in a 30 mL of sodium acetate buffer (100 mM, pH 4.5). This was subsequently dialyzed with the same buffer using a Membrane filter No 110 with 12–14 kDacut off (Hi-Media, India). Later, the dialyzed fraction was loaded on adiethylaminoethyl (DEAE) cellulose resin and then eluted with a linear salt gradient (0–0.8 M sodium chloride) in a sodium acetate buffer (100 mM, pH 4.5), followed by further purification on a Sephadex G-100 column. The active fractions were then pooled and assayed for protein content and enzyme activity [12].

### Characterization of the purified enzyme

#### Determining the molecular weight of the enzyme

The homogeneity and molecular weight of the purified protein fraction were determined using Sodium Dodecyl Sulfate Polyacrylamide Gel Electrophoresis (SDS-PAGE). The purified fractions and standard protein marker (Ge-Nei, Bengaluru, India) were electrophoresed on SDS-PAGE, comprising of a resolving gel (10%) and a stacking gel (5%) [31]. The electrophoresis separated bands were then stained with Coomassie Brilliant Blue R-250. Subsequently, the molecular mass was estimated by comparing the separated bands with the standard protein markers. The protein content of the supernatant at each stage was estimated according to the method of Lowry et al. [32], using bovine serum albumin (1000 μgmL^-1^) as a standard.

#### Determining the protein sequence of the enzyme using MALDI-TOF

The purified enzyme band obtained in the SDS-PAGE gel was excised carefully and was subsequently subjected to trypsin digestion [33]. The digested peptides were analyzed on MALDI-TOF/TOF (Bruker Daltonics, Germany). The peptide mass fingerprint (PMF) analysis was then conductedusing the Flex analysis software. The mass obtained through the PMF was then submitted for the Mascot search in the database for identifying the protein and was later compared with the NCBI-nr database.

### Optimization experiments on purified laccase

#### Influence of pH on enzyme activity and pH stability

The influence of pH on the enzyme activity was investigated by dissolving the substrate (ABTS and guaiacol) in 50 mM glycine-HCl buffer (pH 3.5), citrate phosphate buffer (pH 7.5), and glycine-NaOH buffer (pH 710). Afterbeing incubated at 34 °C, the enzyme activity was measured at 420 nm.

For studying the pH stability of the enzyme, the partially purified enzyme was pre-incubated at various pH ranges (2–10) for 60, 120, and 240 min at 34 °C, followed by the estimation of residual enzyme activity using ABTS substrate.

#### Influence of temperature on enzyme activity and thermal stability

The temperature profile of laccase activity was studied in a1.0 mM ABTS system. The oxidation of ABTS was conducted at various temperatures in the range of 20–80 °C [34]. For studying the thermal stability of the enzyme, it was incubated with 1.0 mM ABTS in the temperature range of 34–75 °C for 150 min. The samples were withdrawn after every 30 min and then estimated for enzyme activity.

#### Influence of inhibitors on laccase activity

Various inhibitors, such as sodium azide (NaN_3_) (0.05–0.30 μmmL^-1^), cysteine (100–400 μmmL^-1^), Ethylenediaminetetraacetic acid (EDTA) (10–100 μmmL^-1^), halides (I-, Cl-, F-) (100–500 μmmL^-1^), thioglycolic acid (500–1500 μmmL^-1^), and thiourea (500–1500 μm mL^-1^) were evaluated to assess their effect. Furthermore,the partially purified enzyme was separately incubatedusing ABTS as the substrate and different concentrations of each inhibitor, for 10 min at 34 °C. The enzyme activity was subsequently determined.

#### Effect of activators (metal ions) on laccase activity

The effect of various metal ions, such as Al^3+^, As^2+^, Ag^2+^, Cd^2+^, CO^2+^, Cu^2+^, FeCl_3_, FeSO_4_, Hg^2+^, Mg^2+^, Mn^2+^, MO^2+^, Ni^2+^, Zn^2+^, and Li^2+^ (1 mM) on the laccase activity was examined by incubating the enzyme along with the metal ions and 1.0 mM ABTS, for 15 min at 34 °C [35]. The residual activity of the enzyme, with a reference enzyme as 100%, was then estimated.

#### Immobilization of the enzyme

The entrapment method was used to immobilizethe laccase, using a 1:1 mixture of 1.5% (w/v) of gelatine and 3.0% (w/v) of sodium alginate. A 1.0 mL purified laccase was added to this mixtureand then thoroughly mixed for 10 min at 25 °C. Afterward, this mixture was withdrawn using a 5 mL sterile syringe, with a 22 gauge needle. This mixture was then extruded into a 2.0% (w/v) pre-chilled CaCl_2_ solution to form the beads, with the diameters of 2.0 to 3.0 mm [36]. The immobilization efficiency was calculated by comparing the enzyme activity of the free enzyme and immobilized enzyme.

### Enzyme kinetics

Kinetics of the laccase were studied using ABTS (10–200 mM) as the substrate. The apparent Km and Vmax values were calculated by Michaelis-Menten and Lineweaver-Burk plot, using Graph Pad Prism 7.0 and Sigma Plot 12.0 software (San Diego, US) applications.

### Evaluating dye decolorization potential of the enzyme

The ability of the immobilized laccase to decolorize various non-textile dyes, viz. methyl red, crystal violet, bromothymol blue, bromophenol blue, bromocresol purple, methylene blue, safranin, and methyl orange, was examined in the presence of 2 mM LMS (1-hydroxy benzotriazole (HBT). The decolorization reaction mixture, containing 50 mL 100 mM sodium acetate buffer (pH 4.5), dye (200 mgL^-1^), and enzyme (0.5 gm immobilized beads equivalent to 5 UmL^-1^), was incubated at 34 °C for 96 h [12]. The degree of dye decolorization was estimated by recording the change in the absorbance at a respective λmax and calculated as percentdecolorization by deducting the control from the absorbance of the sample [37].

### Statistical analysis

All experiments were conducted in triplicate and the results were expressed as mean ± standard error/deviation.

## Result and discussion

### Screening and production of laccase

*Aspergillus* sp. HB_RZ4 was observed to produce brown halos around and under the growth on the GuA plate, indicating the production of ligninolytic enzymes. It oxidized ABTS from ABTS agar and produced a green halo around the mycelia growth,thus, confirming the production of laccase. During submerged fermentation under shaking conditions at 32 °C on the eighth day of incubation,*Aspergillus* sp. HB_RZ4 was found to produce 6.22 UmL^-1^ laccase.

### Optimization of laccase production

#### Influence of incubation period on laccase activity

In the time-course studies, maximum laccase activity (8.422 UmL^-1^) and optimum growth (0.0021 mgmL^-1^) were found to be evident on the eighth day of incubation (Fig 1).

**Fig 1:** Influence of incubation period on laccase production in the basal medium. The samples were withdrawn after every 24 h and were estimated for laccase activity and fungal growth.

#### Influence of pH and temperature on laccase production

The pH and temperature profile of laccase activity revealed that the optimum enzyme activity (8.125 UmL^-1^) was obtained at an acidic pH value of 4.5 and the incubation temperature of 34°C. pH values below and above 4.5 were observed to affect the enzyme activity. Similarly,incubation temperature below or above 34°C was found to affect the growth as well as laccase production.

#### Influence of carbon and nitrogen source on laccase production

Among the various carbon sources used for producing laccase in *Aspergillus* sp. HB_RZ4, glucose was observed to increase the production of laccase by 12.45 times. Furthermore, glycerol containing media were observed to have the lowest laccase yield (2.761 UmL^-1^). The order in which the carbon sources supported laccase production was glucose> sucrose> starch> maltose> lactose> fructose> glycerol. Among the organic and inorganic nitrogen sources, the maximum laccase activity (6.581 UmL^-1^, 11.7 times increase) was obtained with the yeast extract, while ammonium nitrate was found to be the best inorganic nitrogen source as it yielded a laccase activity of 3.97 UmL^-1^ (Table 1).

**Table 1:** Influence of nitrogen sources on the production of laccase in *Aspergillus* sp. HB_RZ4.

Organic nitrogen source	Laccase production (UL^-1^)		Specific activity (Umg^-1^)	Times increase
	In the absence of an inducer	In the presence of an inducer		
L-asparagine	2.55	1.225	30.4	4.79
Glutamic acid	3.96	1.949	32.7	4.92
Glycine	3.84	1.087	26.3	2.83
L-proline	1.58	3.968	78.3	2.51
Yeast extract	5.62	6.581	208.8	11.7
Peptone	4.12	3.951	78.9	9.37
Urea	1.36	4.174	18.5	2.32
NH_4_NO_3_	3.97	2.649	64.0	6.67
NaNO_3_	3.02	1.492	32.5	4.93
KNO_3_	1.69	2.080	11.2	1.23
NH_4_Cl	2.08	0.996	25.7	4.78
NH_4_H_2_PO_4_	3.09	1.277	31.6	4.13
(NH_4_)_2_SO_4_	2.15	0.9621	23.2	4.47

These figures represent the average of triplicates, with a standard deviation of 5%

#### Purification of laccase

Among the various methods used for purification, the best laccase for *Aspergillus* sp. HB_RZ4 was obtained on the Sephadex G-100 column. This method yielded a total protein content of 2.0 mg, enzyme activity of 1.212 U, and specific activity of 465 Umg^-1^ proteins,resulting in a 6.21% purification yield, with 65 times purification. Salt precipitation and DEAE-cellulose methods resulted in minimum protein contents (0.2 and 0.7 mg), low enzyme activities (93 and 105 U), less specific activities (60 and 150 Umg^-1^),poor purification yield (4.73%), and minimum fold purifications (8.5 and 21), respectively, (Table 2).

**Table 2:** Summary of purification of laccase of *Aspergillus* sp. HB_RZ4 by various methods.

Step	Total Protein (mg)	Total activity (U)	Specific activity U/mg	Yield %	Purification fold
(NH_4_)_2_SO_4_ precipitation dialyses	0.2.	93.0	60.95	4.73	8.5
DEAE-cellulose	0.7	105.3	150.4	5.36	21.0
Sephadex G- 100	**2.0**	**121.9**	**465.0**	**6.21**	**65.0**

Figures are an average of triplicates with a standard deviation at 5%

### Characterization of the enzyme

#### Determining the molecular weight

The molecular mass of the purified laccase fraction, as obtained from SDS-PAGE, was found to be approximately 62 kD (Fig 2).

**Fig 2:** SDS-PAGE analysis for the molecular mass of the protein of *Aspergillus* sp. HB_RZ4. Purified fractions of laccase (Lane 2) and standard protein marker (Lane 1) were electrophoresed on SDS-PAGE, followed by staining with Coomassie BrilliantBlue R-250. The molecular mass of purified proteins was estimated by comparing it with the standard protein markers.

#### Determining the protein sequence of the enzyme using MALDI-TOF

Among the various trypsin digested peptide fragments, 10 peptides were hit in the protein database through the Mascot peptide mass fingerprinting search engine. The amino acid sequences of each peptide of the laccase were found to exhibit a significant Mascot score of 75 and a p-value ˂ 0.05 (Fig 3), with a known sequence of NCBI: GAA87354.1. These 10 peptides corresponded to 29.33% sequence coverage and demonstrated homology with the laccase of *Aspergillus kawachii* IFO 4308 (NCBI: GAA87354.1).

**Fig 3:** MALDI-TOF mass spectrum of the trypsin digested peptide map of the laccase. The purified enzyme band obtained in SDS-PAGE was digested by the trypsin and subjected for PMF analysis using the Flex analysis software. The Mascot search in the database and peptide/proteins were compared with the NCBI-nr database.

### Optimization experiments with the purified enzyme

#### Influence of pH on laccase activity and stability

The purified laccase of *Aspergillus* sp HB_RZ4 showed the pH optima of 4.5 and 6.0, with 100% and 99.9% residual activities for ABTS and guaiacol, respectively. The enzyme was found to be stable over a range of pH (neutral to alkaline) for a longer period, i.e., 120 and 240 handhigher stability was evident at neutral pH.

#### Influence of temperature on laccase activity and stability

The enzyme was found to be active over a wide range of temperatures (20–60 °C), with 34 °C being the optimum temperature until 90 min of incubation. Increasing the temperature above 34 °C and incubation period above 90 min was observed to affect the enzyme activity. Good enzymestability (97%) was obtained at 34 °C after 90 min.

#### Influence of inhibitors and activator (metal ions) on laccase activity

Experiments on the influence of different concentrations of inhibitors and metal ions revealed that some inhibitors affected the enzyme activity even at lower concentrations, while others did not affect it, even at relatively higher concentrations. Sodium azidewas observed to completely inhibit the enzyme activity at 0.30 μmmL^-1^, whereas L-cysteine was observed to not affect the enzyme activityeven at a higher concentration (400 μmmL^-1^). While halides were found to strongly inhibit the enzyme, fluoride caused 98.72% inhibition, even at a lower concentration (25 μmmL^-1^). Chloride, bromide, and iodide (300 μmmL^-1^) were observed to cause 96.12%, 94%, and 94.12% inhibition, respectively. Thioglycolic acid was observed to produce strong inhibition (97.10%) than thiourea (91.55%).

Other metal ions, such as Al^3+^, As^2+^, Cd^2+^, CO^2+^, and Li^2+^,were observed to significantly inhibit the activity of the enzyme, while Ag^2+^, Hg, FeSO_4_, and FeCl_3_ demonstrated 90%, 95%, 78%, and 76% inhibition, respectively. Cu^2+^, Mo^2+^, Mn^2+^, and Zn^2+^ were found to be enhance the enzyme activity. The presence of Cu^2+^ was observed to significantly boost the enzyme activity from 8.125 to 8.692 UmL^-1^ (Fig 4), whereas, vanillin, ammonium tartrate gallic acid, and vanillic acid failed to enhance the enzyme, however, they were observed to affect the enzymeactivity. A 25 μM CuSO_4_ was observed as the threshold level for the optimum laccase activity and fungal growth (8.692 UmL^-1^, 0.019 mgmL^-1^).

**Fig 4:** Influence of various concentrations of CuSO_4_ on the laccase activity. The reaction mixture contained the enzyme, along with CuSO_4_ (0–50 μM), for 15 min at 34 °C. The enzyme activity was measured with 1.0 mM ABTS, keeping reference enzyme as 100%.

#### Evaluating dye decolorization potential of the enzyme

The LMS was observed to have negligible effect on the dye decolorization potential of laccase, and the absence of LMS resulted in 86%, 92%, 98%, and 95% decolorization of the bromothymol blue, methyl red, bromophenol blue, and bromocresol purple, respectively. Contrarily, the presence of LMS was observed to inhibit the decolorization of methyl red, safranin, and methyl orange. However, forcongo red, crystal violet, and methylene blue,the LMS was observed to increase the decolorization of these dyes by 1.49, 1.99, and 3.47 times, respectively.

### Enzyme immobilization

The immobilized enzyme was observed to exhibit 92% enzyme efficiency (8.556 UmL^-1^) vis-à-vis 100% efficiency (9.30 UmL^-1^) of the free enzyme and it was observed to deteriorate with increasing period. On the eighthday,the incubation enzyme efficiency was observed to reduce to 48.38% (4.5 UmL^-1^).

### Enzyme kinetics

The kinetic parameters Km and Vmax of the purified laccase were found to be 26.8 mM and 7132.6 mMmin^-1^, respectively.

## Discussion

Fungi are the most widespread saprophytes that degrade organic matter by secreting manylignolytic enzymes, including laccase. Formation of brown halos around and under the growth of *Aspergillus* sp. HB_RZ4 on the GuA plate was due to the oxidation of guaiacol,indicating the production of lignolytic enzymes. The formation of green halo around the mycelia growth was due to the oxidation of ABTS (substrate) to a stable colored product, 2,2’-azino-bis(3-ethylbenzothiazoline-6-sulfonate), under the influence of laccase [38]. Since ABTS was a specific substrate for laccase, its oxidation indicated that the enzyme produced by *Aspergillus* sp. HB_RZ4 was a pure laccase [24]. Bothof these screening tests confirmed the ability of *Aspergillus* sp. HB_RZ4 to produce laccase. It produced 6.22 UmL^-1^ laccase on the eighth day of incubation during the shake flask growth at 32°C. Ghosh and Ghosh [39] reported more laccase production from *A*. *flavus* on the twentieth day of incubation. Kumar et al. [24] reported optimum laccase production (17.39 IUmL^-1^) in *A*. *flavus* on the twelfth day of incubation. Some fungal species require longer production time, i.e., 12–30 d [39]. Sivakumar et al. [40] reported a 4.60 IUmL^-1^ laccase yield after 12 d of incubation under static conditions. In many fungi, laccase synthesis is activated by the type and nature of carbon or nitrogen source, which determines the duration of the production cycle. Therefore, it was considered that the best laccase producing organism should produce high yields of laccase in a short fermentation cycle [41]. A higher yield of laccase in less time (8 d) reflects the metabolic efficiency of the organisms and suggests the possibility of exploitingthe organism for cost-effective production of laccase at commercial scale. The optimization of physicochemical parameters was observed to boost the enzyme yield. Optimum laccase yield in glucose and yeast extract containing medium was due to the rapid assimilation of glucose, as it isa readily oxidizable sugar and yeast extract is the source of all amino acids required for the synthesis of laccase [42]. Senthivelan et al. [43] reported the production of laccase in *Penicillium chrysogenum*. The statistical optimization was observed to enhance the enzyme activity to 7.9 UmL^-1^ against 6.0 UmL^-1^ obtained under un-optimized conditions. Laccase production in many fungi, including *P*. *chrysogenum*, was reported to have acidic pH at mesophilic temperature. Media composition, presence or absence of the metal ions, and types and levels of the nutrients have been known to regulate the expression of laccase isozyme genes. The effects of organic compounds on laccase production depend on the compound structure, fungal strain, and growth stage [44]. Fewer purification yields, with ammonium sulfate precipitation, may be due to the denaturation of the enzyme by ammonium sulfate. Furthermore, no purification with DEAE-cellulose may be due to the ability of enzymes to get absorbed on the cellulose matrix. Additionally, good purification yields, with Sephadex G-100 column, can be attributed to better adsorption of enzyme on Sephadex gel. In previous studies, many fungal laccases were purified using Sephadex G-100 resins. Kumar et al. [24] reported the purification of laccase of *A*.*flavus* on Sephadex G-100 resin. Patel and Gupte [45] reported the purification of laccase of *Trichoderma giganteum* AGHP using Sephadex G-75 and found an enzyme yield of 10.49% with 3.33 times purification. A 70-times purification of laccase from *StereumOstrea*, using ammonium sulfate precipitation followed by Sephadex G-100 column chromatography was reported by Vishwanath et al. [46]. The molecular weight of purified laccase of *Aspergillus* sp. HB_RZ4 was found to be 62 k, as evident from the SDS-PAGE gel stained by coomassie brilliant blue (Fig 3). The molecular weight of the fungus resembled the molecular weight of laccases, as reported for other white-rot fungi [47]. Patel and Gupte [45] found the molecular weight to be 66 kDa, using SDS-PAGE. Laccase purified by Sephadex G-100 has been observed to display good specific activity compared to laccase from *Trametes versicolor* [48]. Good activity and stability of the enzyme for longer periods, at wider pH (acidic to alkaline) and temperature ranges (20–60 °C) was due to the presence of specific substrates, such as ABTS and guaiacol. Kumar et al. [24] reported good laccase activity over awide range of pH and temperature in *A*. *flavus*. In this study, the inhibitory effect of sodium azide, cysteine, EDTA, halogens, thioglycolic acid, and thiourea on laccase activity was examined. A drastic decrease in enzyme activity was considered to be due to a change in the pH of the medium that exertedan inhibitory action on the enzyme activity [49]. Severe reduction in the enzyme activity by sodium azide and cysteine was due to the binding of sodium azideat the copper site of the enzyme,which blocked the internal electron transfer reaction. Laccases are sensitive towards metals, even at low concentrations and inhibit the laccase activity. Good induction of enzyme activity in the presence of CuSO_4_ was due to the filling of type-2 copper-binding sites with copper ions and Cu^2+^ being the main inducer for laccase [50], as the catalytic center of the enzyme contained Cu^2+^ ions. Xin and Geng [51] also observed copper sulfateto be the best inducer for laccase production in *Trametes versicolor*. Mann et al. [52] reported 0.75 and 0.4 mM concentrations of copper as the best levels to induce laccase production in *Ganoderma lucidum*. Inhibition of laccase activity at above 25 μM of CuSO_4_ may be because higher concentration of copper has been observed to inhibit the growth of fungi [53]. Potent inhibition of the enzyme activity by Ag^2+^ and Hg^2+^ was attributed to the formation of sulfhydryl (SH) groups with the enzyme, thus, inactivating the enzyme. Moreover, these enzymes are known to possess antimicrobial activity [54]. This interaction of enzyme with the metals has great significance for better understanding and development of a process for bioremediation of xenobiotics, textile dyes, and grey-water. The effect of metal ions on laccase activity depended upon the type of metals used,as the metal ions significantly influenced the catalytic activity of the enzyme. The activation or inhibition of the enzymes also regulated the turnover rate of the enzymes. The enzyme was able to decolorize approximately 88%, 96%, and 99% of bromothymol blue, bromocresol purple, and bromophenol blue, respectively, in the presence of HBT. Copete et al. [55] reported 15% to 40% decolorization of various dyes by laccase producing *Leptosphaerulina* sp. and found enhanced decolorization in the presence of a mediator. Zuo et al. [13] reported 84.9% decolorization of bromocresol by *Pleurotusostreatus* HAUCC 162 and noted the effect of mediator HBT in increasing the decolorization. Enzymes immobilization has been observed to make the enzymes reusable, provide more stability and resistance under diverse conditions, and improve the catalytic activity of laccases [24]. Fungal laccases typically have 3 to 10 glycosylation sites, and 10% to 50% of their molecular weight has been attributed to glycosylation and deglycosylation of laccase has been observed to affect its enzyme kinetics [56]. In this study, after SDS-PAGE electrophoresis, a band excised from the gel was used for identification using MALDI_TOF analysis. The band at ~ 62 kDa was digested with trypsin into 10 amino acid sequence fragments, rangingfrom P1 to P10 (22 to 250 amino acid sequence) (Tables 3 and 4). The Mascot database was found to exhibit 29.33% resemblance with laccase of *A*. *kawachii* IFO 4308 (NCBI: GAA87354.1), which confirmed that the purified enzyme was laccase [57]. Km and Vmax of the purified laccase were found to be 26.8 mM and 7132.6 mMmin^-1^, respectively, which indicated good activity of the enzyme. Tinoco et al. [58] reported the Km values rangingfrom 8 to 79 μmol for ABTS with different strains of *Pleurotusostreatus*.

**Table 3:** Peptide ions of trypsin digest of laccase of *Aspergillus* sp.HB_RZ4.

Designated peptides*	Amino acid sequence of identified peptides			[M+H]^+^		Total number of sequenced amino acids
	Position		Peptide sequence	Observed	Calculated	
	From	To		m/z		
P1	22	33	VSVTNHLEEEPI	175.621	174.436	12
P2	161	170	NEPVPDSLL	277.908	276.645	09
P3	123	139	KDILLLVGDWYHRSADQ	492.263	491.341	17
P4	406	420	GHPFHMHGHHFYILR	563.258	562.463	15
P5	221	240	TLIQVDNIDVEQQDSNSAGV	605.345	604.621	20
P6	451	470	RTDSPYDLSRAQLRDTVYIP	720.306	719.285	20
P7	315	336	LLSGLPAKAHQTHVVYTKIEKL	850.211	849.348	22
P8	273	286	YPNPALASIQTFDI	1006.636	1005.589	14
P9	427	439	GWGAYNPFTDAHP	1017.703	1016.562	13
P10	242	250	YPGQRMDIMLRPSPDETPS	1063.581	1062.354	19

* Peptides of laccase designated from P1 to P10.

**Table 4:** Amino acid content of sequenced peptides of laccase obtained by trypsin digestion.

Amino acid	The number of amino acids per peptide of hyaluronidase*										
	P1	P2	P3	P4	P5	P6	P7	P8	P9	P10	Total
Gly (**G**)	-	-	1	2	1	-	1	-	2	1	08
Ala (**A**)	-	-	1	-	1	1	2	2	2	-	09
Val (**V**)	2	1	1	-	3	1	2	-	-	-	10
Leu (**L**)	1	2	3	1	1	2	4	1	-	1	16
Ile (**I**)	1	-	1	1	2	1	1	2	-	1	10
Ser (**S**)	1	1	1	-	2	2	1	1	-	2	11
Thr (**T**)	1	-	-	-	1	2	2	1	1	1	09
Cys (**C**)	-	-	-	-	-	-	-	-	-	-	00
Met (**M**)	-	-	-	1	-	-	-	-	-	2	03
Asp (**D**)	-	1	3	-	3	3	-	1	1	2	14
Asn (**N**)	1	1	-	-	2	-	-	1	1	-	06
Glu (**E**)	3	1	-	-	1	-	1	-	-	1	07
Gln (**Q**)	-	-	1	-	3	1	1	1	-	1	08
Phe (**F**)	-	-	w-	2	-	-	-	1	1	-	04
Tyr (**Y**)	-	-	1	1	-	2	1	1	1	1	08
Trp (**W**)	-	-	1	-	-	-	-	-	1	-	02
Lys (**K**)	-	-	1	-	-	-	3	-	-	-	04
Arg (**R**)	-	-	1	1	-	3	-	-	-	2	07
His (**H**)	1	-	1	5	-	-	2	-	1	-	10
Pro (**P**)	1	2	-	1	-	2	1	2	2	4	15
**Total**	**12**	**09**	**17**	**15**	**20**	**20**	**22**	**14**	**13**	**19**	**161**

## Conclusion

In this study, *Aspergillus* sp. HB_RZ4 produced copious amounts of extracellular laccase in MM under mesophilic conditions at acidic pH. The conventional inhibitors and chemicals used in the present study did not inhibit the production of laccase. The stability of laccase over the range of pH and temperature and the ability to decolorize the dye without requiring LMS makes it a magic molecule due toits cost-effective production and its usage in bioremediation of effluent containing dyes.

## Supporting information

S1 Fig (TIF)
